# CXR-RefineDet: Single-Shot Refinement Neural Network for Chest X-Ray Radiograph Based on Multiple Lesions Detection

**DOI:** 10.1155/2022/4182191

**Published:** 2022-01-07

**Authors:** Cong Lin, Yongbin Zheng, Xiuchun Xiao, Jialun Lin

**Affiliations:** ^1^College of Electronics and Information Engineering, Guangdong Ocean University, Zhanjiang 524025, China; ^2^College of Biomedical Information and Engineering, Hainan Medical University, Haikou 571199, China

## Abstract

The workload of radiologists has dramatically increased in the context of the COVID-19 pandemic, causing misdiagnosis and missed diagnosis of diseases. The use of artificial intelligence technology can assist doctors in locating and identifying lesions in medical images. In order to improve the accuracy of disease diagnosis in medical imaging, we propose a lung disease detection neural network that is superior to the current mainstream object detection model in this paper. By combining the advantages of RepVGG block and Resblock in information fusion and information extraction, we design a backbone RRNet with few parameters and strong feature extraction capabilities. After that, we propose a structure called Information Reuse, which can solve the problem of low utilization of the original network output features by connecting the normalized features back to the network. Combining the network of RRNet and the improved RefineDet, we propose the overall network which was called CXR-RefineDet. Through a large number of experiments on the largest public lung chest radiograph detection dataset VinDr-CXR, it is found that the detection accuracy and inference speed of CXR-RefineDet have reached 0.1686 mAP and 6.8 fps, respectively, which is better than the two-stage object detection algorithm using a strong backbone like ResNet-50 and ResNet-101. In addition, the fast reasoning speed of CXR-RefineDet also provides the possibility for the actual implementation of the computer-aided diagnosis system.

## 1. Introduction

Chest X-ray (CXR) is an effective and widely used imaging technique in the diagnosis and screening of lung-related diseases. The imaging principle and structure of chest radiographs are complex, which requires professional radiologists to spend a lot of time to observe carefully. Medical research [1, 2] shows that postprocessing of medical images by using a computer-aided diagnosis (CAD) system can effectively reduce the initial screening of chest radiographs and improve the accuracy of lesion screening. Benefiting from the rapid development of the field of artificial intelligence [3], many researchers have proposed lots of automatic diagnosis methods by combining deep learning technology with imaging examination technology to reduce the workload of radiologists and the possibility of misdiagnosis [4, 5]. The use of deep learning technology to assist doctors in diagnosing diseases has become a new trend.

The application of deep learning in the field of medical imaging is mainly in the two major tasks of segmentation and detection. Because of the reason that the segmentation task can provide doctors with precise lesion area positions and is more suitable for actual needs, it has become a research hotspot in the field of medical imaging [6, 7]. Arnaud proposed a new computer-aided detection lung nodule system using multiview convolutional networks (ConvNets) to reduce the false positives of the CAD system [8]. Olaf proposed a segmentation network U-Net [9] that efficiently utilizes medical image annotation, which vigorously promotes the development of medical image segmentation. Rocha [10] proposed a lung nodule segmentation method based on U-Net and SegU-Net to solve the segmentation problem of lung nodules in computed tomography. The segmentation results of lung nodules by this method can help doctors further analyze the lesions feature. However, the segmentation model may be inaccurate for the segmentation of the edge part of the lesion and the small lesion area in practical applications since the spatial dimension of a chest X-ray is usually 2000 × 3000 pixels and the local lesion area is relatively small, which makes the detection more difficult and requires the doctor to spend more time to make further judgments.

Different from image segmentation, object detection provides a candidate area of the lesion, which will help the doctor to quickly locate the lesion area instead of focusing on the pixel-level segmentation area [11]. In terms of lung disease screening, studies [12–15] have shown that detection models designed through deep learning can provide doctors with areas where lung disease may occur, which can greatly improve the efficiency of disease screening by radiologists. In order to detect the location, type, and attributes of lung lesions more accurately, Yan designed a deep learning module that extracts relevant semantic tags from radiology reports related to lesion images. Using image and text to mine tags, a lesion annotation network (LesaNet) based on multilabel convolutional neural network is proposed to learn all the tags in a comprehensive way [16]. Liang proposed a method to filter out target images with lung nodules from the patient's whole lung CT images by training a classification network and then use Faster RCNN to detect the location range of the suspected lung nodules in the CT image to increase the reliability of the detection and reduce the false positives of detectors [17]. Xiao [18] proposed a fully automatic lung nodule detection algorithm using a cascade strategy based on FPN [19]. By designing multiple stages of detection networks and integrating them into a heterogeneous classification network, the nodules are gradually separated from the lung background. Although the lung lesion detection methods based on the two-stage object detection model have higher detection accuracy, the two-stage object detection model is larger and occupies high computing resources, and it is difficult to deploy to the detection system of the hospital. Therefore, most of the current lesion detection models of medical images tend to use a combination of one-stage object detection algorithms and large backbone, such as using RetinaNet [20] as the base model and matching large backbone such as ResNet-101 [21] and SE-ResNet-101 [22] to detect lung lesions. Although this can increase the detection accuracy while speeding up the detection speed, these base models still require high computing resources and cannot be well applied in medical auxiliary detection systems.

From the above analysis, it can be seen that the high requirements of computing resources, slow reasoning speed, and low accuracy of detecting lesions hinder the application of artificial intelligence technology in the field of medical images. In order to solve the above problems and promote the implementation of computer-aided diagnosis technology in chest radiography, a chest radiograph lesion detection algorithm with a small model, high accuracy, and fast detection speed based on RefineDet network architecture is proposed in this paper. In the first step, we designed a backbone RRNet with a small amount of parameters and strong feature extraction capabilities by combining the advantages of RepVGG block and Resblock in information fusion and information extraction, which can improve the feature extraction capabilities of the network while reducing the amount of model calculations. Then, we proposed a structure called Information Reuse through connecting the normalized features of RefineDet back to the network again, which can effectively solve the problem of low utilization of the original network output features and achieve the purpose of improving detection accuracy. Combining the network of RRNet and the improved RefineDet, we propose the overall network named CXR-RefineDet. A large number of experiments have been done to verify the performance of CXR-RefineDet on VinDr-CXR [23], and the experimental results show that the RRNet backbone and Information Reuse structure we designed have brought about 0.99% and 0.72% improvement in detection performance, respectively. In addition, we also compare with the current mainstream object detection network on the three performance indicators of mAP, inference speed, and parameter amount. As shown in Figure 1, the comparative experiment results show that the detection accuracy and speed of the CXR-RefineDet network greatly exceed the existing mainstream object detectors under the condition of moderate parameter amount, which can effectively help doctors quickly and accurately screen the location of lesions in the image.

The main contributions of this work are as follows: (1) By combining the advantages of RepVGG block and Resblock in information extraction and information fusion, we designed a backbone RRNet with few parameters and strong feature extraction capabilities. (2) We propose the Information Reuse structure, which solves the problem of low utilization of the original network output features by linking the normalized features back to the network. (3) The proposed object detection model CXR-RefineDet has a good performance between accuracy and speed. It achieves 0.1686 mAP and 6.8 fps on the VinDr-CXR dataset, which is significantly better than mainstream object detection models.

## 2. Materials and Methods

### 2.1. Related Works

The one-stage object detection network RefineDet [24] proposed by Zhang adds Anchor Refinement Module (ARM) and Object Detection Module (ODM) to the network to perform preliminary filtering and further filtering of anchor frames, respectively. At the same time, the network also uses the Transfer Connection Block (TCB) module to fuse the features between ARM and ODM, so that the one-stage object detection network has the accuracy of the two-stage object detection network while maintaining a faster detection speed, which could make it possible for the model to be implemented. It should be pointed out that the backbone of RefineDet has two types, VGG-16 [25] and ResNet-101, but ResNet-101 has a large amount of parameters and requires high computing resources. Compared with ResNet-101 which stacks more residual blocks, VGGnet has the advantages of fewer network parameters and faster running speed. Considering that the efficiency of the medical auxiliary detection system is more important in practical applications, choosing VGG-16 as the backbone of RefineDet for medical image detection will be more practical. The contribution of VGG-16 proposed by Karen is a thorough evaluation of networks of increasing depth using an architecture with very small convolution filters, which shows that a significant improvement on the prior-art configurations can be achieved by pushing the depth to 16–19 weight layers [25]. Recently, many researchers have proposed excellent variant networks based on VGG. Huang [26] connected the low-level semantic information of the network with many high-level semantic information to build a complex network topology Densenet. Inspired by the ResNet and Inception structures, [27] designed the ResNext network structure by adding residual connections to the Inception structure. Zhang constructed the ResNeSt [28] network by introducing the Split Attention module and SKNet-block [29] on the basis of ResNeXt. Although new network structures are emerging one after another and the accuracy of the network has also been greatly improved, the amount of network parameters and requirements for computing resources have also become higher and higher. In addition, various new network module functions are complicated to implement, which further aggravates the difficulty of model deployment.

### 2.2. Network Architecture

In the previous analysis, it was mentioned that ResNet-101 needs to consume more computing resources, and the residual structure in ResNet requires that the feature dimensions before and after the residual must match, which limits the flexibility of the network, so we chose VGG-16 as the backbone of RefineDet. At the same time, we noticed that the RepVGG [30] network proposed by Ding is only composed of 3 × 3 convolution, BN layer, and ReLU modules, which is very beneficial to the acceleration of the neural network of mobile devices. In addition, since Resblock can fuse the feature information between multiple convolutional layers through jump connections between layers, and RepVGG block can improve the feature extraction ability of single-layer convolution after paralleling multiple convolution modules in a single convolution layer, we believe that combining the advantages of RepVGG block and Resblock in single-layer convolution and multilayer convolution can greatly improve the detection ability of the backbone. Considering that the network shallow convolution is responsible for extracting low-level semantic features, and the information richness of this part of the low-level semantic features directly determines the effectiveness of the high-level semantic features of the subsequent convolutional layer, we set the first three layers of the new backbone named RRnet as RepVGG block and use the feature of multiple modules in parallel to improve the information extraction ability of the network's shallow convolution, while the remaining layers are set as Resblock modules to fuse high-level semantic features between cross-layer convolutions. In addition, we found that the features of the first two network output layers after L2 normalization in RefineDet have not been effectively used, which reduces the detection capabilities of the latter two network output layers. In order to solve this problem, we designed the Information Reuse structure to connect the first two network output layers to the network again through the characteristics of L2 normalization. Combining the backbone RRNet we designed and the improved RefineDet network architecture, we finally got the new object detection model CXR-RefineDet, which is shown in Figure 2.

It can be seen from Figure 2 that CXR-RefineDet introduces three modules of ARM, ODM, and TCB of RefineDet network to improve the detection performance of the network. The role of the ODM module is to further accurately determine the position of the anchor frame and predict the category information of the anchor frame. The TCB module exists between the ARM and ODM modules; it integrates the context information to a greater extent by transferring the characteristics of the ARM modules in different output layers to the corresponding ODM module to improve the detection capability of the ODM module. The new backbone RRnet is designed by integrating the structure of Resblock and RepVGG block to solve the problem of poor information extraction ability of the original backbone. The structure of RRNet and Information Reuse will be further discussed in next sections.

Many natural image processing methods in computer vision have strongly relied on ImageNet pretrained deep CNN models [31] so far. These models have performed well in a large number of object categories and provide a good baseline for further model fine-tuning. In the field of object detection, the backbone usually uses a pretrained model for migration learning, which can accelerate the convergence speed of the network while improving the detection accuracy of the network. However, the use of pretraining models limits the flexibility of the network structure. Existing pretraining models are based on specific network structures such as ResNet-50 and ResNet-101, and their computing resource consumption often cannot meet the requirements of edge computing systems. In addition, pretraining models may not be suitable for the field of medical image diagnosis since the medical images are quite different from traditional RGB images. Using ImageNet pretraining models may cause domain mismatch problems, while training the network from scratch can avoid these problems. In summary, we follow the settings in ScratchDet [32] and introduce the BatchNorm layer in the RefineDet network, while using a larger learning rate for training.

### 2.3. New Design Backbone

To solve the problems of gradient dispersion and gradient explosion in deep neural network training, the residual structure proposed of ResNet introduced the jump connections in stacked convolution modules, as shown in Figure 3(b). The introduction of residual connections can fuse the feature information between different network layers, which is very beneficial for the detection of medical images. As we know, the neural network extraction of image information is a process from shallow to deep [33]. The size of the feature map will decrease as the number of network layers deepens, and the deeper the number of network layers, the more delicate the semantic information contained in the feature map. Therefore, the residual connection can further merge the fine-grained features between different convolutional layers. For example, the position of the heart and the lung lobes are included in the lung X-ray image, so the disease of cardiac hypertrophy includes the texture of the lung lobes, and the residual connection can correlate this part of the characteristic information well.

In addition, the introduction of the residual connection will not increase the model parameters since the residual connection is only the summation operation of the feature information between different network layers. As shown in Figure 3(a), unlike the cross-layer information fusion in ResNet, the multibranch topology of RepVGG is paralleled with 1 × 1 convolution (additional BN layer) and BN layer on both sides of 3 × 3 convolution (additional BN layer). Through summing the feature information extracted by different convolution modules, the information extraction capability of a single convolution module can be improved.

In our opinion, Resblock belongs to cross-layer information fusion since it merges fine-grained features between different layers through jump connections between layers. The RepVGG block connects multiple convolutional layers in parallel on a single convolution module to enrich the feature information contained in the single-layer convolution, which belongs to information fusion within the layer. Therefore, we combined Resblock and RepVGG block to design a new backbone RRNet, which can improve the information extraction capabilities of the backbone in single-layer convolution and cross-layer convolution. The network structure is shown in Figure 4(b).

The network shallow convolution is responsible for extracting low-level semantic features such as grayscale and texture, and the information richness of this part of the low-level semantic features directly determines the effectiveness of the high-level semantic features of the subsequent convolutional layer. With this in mind, we set the first three layers of the network as RepVGG block and use the feature of multiple modules in parallel to improve the information extraction ability of the network's shallow convolution, while the remaining layers are set as Resblock modules to fuse high-level semantic features between cross-layer convolutions. The backbone RRNet we designed has fewer network layers and higher accuracy than ResNet-34.

### 2.4. The Architecture of Information Reuse

We follow the settings in RefineDet and select four convolutional layers (Conv4_3, Conv5_3, Conv6_1, and Conv6_2) of different sizes in the backbone as the output of the network, as shown in Figure 5. Conv4_3 and Conv5_3 pass through L2 normalization as the first two outputs of the network, and Conv6_1 and Conv6_2 add two additional convolutional layers at the end of the VGG-16 network as the last two outputs of the network.

Although L2 normalization is added to con4_3 and conv5_3 to scale the feature norms, the scaled features are not further utilized in subsequent networks, so only the object detection effects of the first two networks output feature maps *x*_1_ and *x*_2_ have been improved. The structural information in the image is continuous in space and time. The shallow features extracted by the network are the representation of the deep features of the image. Using the shallow feature information extracted at the beginning of the network will help to improve the effectiveness of the subsequent extraction of deep features. Therefore, we connect con4_3 and conv5_3 to the network again after the scaling feature of L2 normalization, as shown in Figure 5. After this operation, the subsequent neural network can obtain the scaling characteristics of the output layers of the first two networks, which can improve the detection capability of the overall network.

## 3. Results and Discussion

### 3.1. VinDr-CXR Dataset

In order to learn to annotate lesions, a large-scale and diverse lesion image dataset is required. Existing lesion datasets are usually either too small or insufficiently diverse. Fortunately, the recently released dataset VinDr-CXR greatly alleviates this limitation. VinDr-CXR is a chest radiograph dataset released by Vingroup Big Data Institute (VinBigdata) that has the most local labels and the richest number of categories so far. VinBigdata collected more than 100,000 chest radiographs from two major hospitals in Vietnam and invited 17 professional radiologists to manually label 18,000 images, of which 22 types of lesions are local tags and 6 types of special lesions are global label. In addition, VinDr-CXR dataset is divided into 15,000 training sets and 3000 test sets. The images in the training set are independently annotated by 3 doctors, and the images in the test set are jointly annotated by 5 doctors. Since 8 of the 22 categories containing local location information have a small number of images, we merge these 8 smaller categories into other lesions, and then our task is finally defined as an object detection problem for 14 types of lesions, which includes (1) aortic enlargement, (2) atelectasis, (3) calcification, (4) cardiomegaly, (5) consolidation, (6) interstitial lung disease (ILD), (7) infiltration, (8) lung opacity, (9) nodule/mass, (10) other lesions, (11) pleural effusion, (12) pleural thickening, (13) pneumothorax, and (14) pulmonary fibrosis. The distribution of each lesion category is shown in Figure 6.

### 3.2. Training Settings

Because the imaging principle of natural image is very different from that of medical image, the application effect of the pretraining model in medical image is not as good as the model trained from scratch. Therefore, we adopt the pretraining model and the corresponding parameter settings are fine-tuned according to ScratchDet and the experimental results, whose earning rate is 0.05, using SGD with 0.0005 weight decay and 0.9 momentum. Other training strategies mostly follow RefineDet, including data augmentation, hard negative mining, scale and aspect ratios for default boxes, and loss functions. All conv-layers are initialized with the xavier uniform method. The training of other networks such as Reitinanet and Faster RCNN is based on the mmdetection framework, and the Imagenet pretraining model and default parameters are used for training.

### 3.3. Ablation Study

In order to verify the effectiveness of the backbone RRNet and Information Reuse structure, we conduct ablation experiments on VinDr-CXR. In addition, we conducted comparative experiments on mainstream object detection models and compared the performance of various parameters of the models to prove the superiority of the proposed model. Specifically, we resize all the images in the training set to 512 × 512 resolution, but the test set is not resized, and the relevant hyperparameters for model training are kept consistent to ensure a fair comparison. All models are trained and tested on the official training set and test set and submitted to the official platform for result evaluation. The detection results were evaluated using standard PASCAL VOC 2010 [34] mean Average Precision (mAP) at IoU > 0.4.

### 3.4. RRnet

We did two comparative experiments to validate the effectiveness of our new design backbone. A comparative experiment is to replace all layers of VGG-16 with Resblock and RepVGG block, and the other is to replace with two different depths of ResNet and four different versions of RepVGGnet VGG-16, as shown in Table 1. The experimental results in the first row of Table 1 show that the number of layers of the backbone RRNet we designed is less than that of ResNet-34, but the accuracy is 0.47% higher. This proves that, in our analysis in Section 2.3, the information fusion of the Resblock and RepVGG block modules in the cross-layer convolution and single-layer convolution modules can well correlate the characteristics of the lesions, thereby improving the ability of the network to extract feature information. We use Resblock and RepVGG block to replace all layers of VGG-16 and name them All-Resblock and All-RepVGG block, respectively. The two backbones obtained accuracy of 0.1521 and 0.1513, respectively, which are both higher than the ResNet-18 backbone, and the performance is equivalent to that of the ResNet-34 backbone, which verifies the effectiveness of the two modules.

In addition, it can be seen from Table 1 that the accuracy values of RepVGG-A0, A1, RepVGG-B0, and B1 are 0.1374, 0.1409, 0.1434, and 0.1488, respectively, which are lower than the accuracy value of directly replacing all layers of VGG-16 with RepVGG block. The reason is that although the RepVGG series backbones all include RepVGG block, their network tasks are designed for classification, so the difference between tasks causes the performance of the network to deteriorate. The backbone RRnet with 0.1572 mAP is higher than all versions of the backbone, which proves the effectiveness of RRnet.

### 3.5. Information Reuse

To demonstrate the effectiveness of the Information Reuse in the network, we use the network connection output in the original RefineDet and our improved information reuse structure for comparative experiments, whose results are shown in the second and third columns of Table 2. After adding an improved Information Reuse structure to the basic network, the mAP is 0.1587. Compared with the basic network, adding the Information Reuse structure can bring an improvement of 0.72% mAP to the detector, which proves that reconnecting the zoom feature of the network output layer to the network through the Information Reuse structure can improve the performance of the detector.

### 3.6. Network Performance

In order to prove the superiority of the model, we use the three performance indicators of mAP, inference speed, and parameter quantity to conduct comparative experiments on the mainstream object detection model, and the experimental results are shown in Table 3. Compared with large-scale backbone networks such as ResNet-50 and ResNet-101, the model RefineDet with VGG-16 backbone greatly exceeds other mainstream object detectors in detection speed. The low-resolution version with 320 × 320 size of RefineDet has a detection speed of 10.8 fps, and the high-resolution version with 512 × 512 size has a detection speed of 9.9 fps. However, the low-resolution and high-resolution detection speeds of CXR-RefineDet using RRNet as the backbone are 9.6 fps and 6.8 fps, respectively.

In terms of detection accuracy, the low-resolution version of CXR-RefineDet obtained 0.1392 mAP, which surpassed RetinaNet with ResNet-50 backbone. The high-resolution version with 512 × 512 size of CXR-RefineDet obtained the highest detection accuracy of 0.1686 mAP. Compared with the multistage object detection algorithm Cascade RCNN, the model parameters of CXR-RefineDet are smaller than its backbone (ResNet-50, ResNet-101), and the accuracy is better than all its submodels. We also compare with the classic two-stage object detection algorithms Faster RCNN and GA-Faster RCNN. Although the model parameters of CXR-RefineDet with ResNet-101 backbone are slightly higher, it achieves better results in terms of detection accuracy and inference speed. In addition, we have also conducted comparative experiments with anchor-free object detection methods. VFNet [35] and ATSS [36] based on ResNet-101 backbone are slightly higher than CXR-RefineDet in model parameters, but CXR-RefineDet is better than the two methods in terms of speed and accuracy.

Based on the analysis of the above experimental results, it can be seen that the backbone RRNet and Information Reuse structure can effectively improve the detection accuracy of the network. Compared with the use of ResNet-50 and ResNet-101 as the object detector of the backbone, CXR-RefineDet not only has fewer parameters but also can reach a higher and faster level in detection accuracy and speed.

### 3.7. Analysis of Lesion Detection Results

The comparison diagram of detection results between RefineDet and improved CXR-RefineDet network is shown in Figure 7. It can be seen that the detection effect of CXR-RefineDet is better than that of RefineDet network. In the detection results of the first and third rows, RefineDet cannot detect the lesions on the edge of the lung, and its detection performance is also poor for large lesions such as spine distortion. The detection result of CXR-RefineDet is similar to the truth box, and there is no missed detection or false detection. For the detection of some small targets, the detection results in the second row show that the detection rate of small targets of CXR-RefineDet is much higher than that of RefineDet. However, due to the small input resolution with 512 × 512, some smaller lesion areas may also be missed. For some lesions that are both small targets and extreme aspect ratios, RefineDet and CXR-RefineDet have low detection rates for these lesions, such as the red true target box in the lower left corner of the fourth row. Because the imaging principle of medical image is more complex, it does not have better discrimination than natural image. Moreover, due to the equipment, it is easy to be doped with noise in the imaging process, which brings great difficulties to the image detection. For areas with small lesions, even experienced doctors need a long time to distinguish them through naked eye observation. In addition, in order to reduce the complexity of the model, the proposed network model has fewer layers and smaller parameters, which limits the improvement of model detection ability.

## 4. Conclusions

In order to solve the problem of weak feature extraction capability of the RefineDet backbone network and low feature utilization of the output feature layer, a high-precision and fast detection speed lung lesion detection network CXR-RefineDet is proposed in this paper. By combining the advantages of RepVGG block and Resblock in single-layer and multilayer convolution modules, we designed an efficient backbone which was named RRNet. In view of the situation that the original network output features are not used, we introduce the Information Reuse structure to reconnect the features of the network output layer back to the network to improve the detection ability of the subsequent network. CXR-RefineDet is tested on VinDr-CXR dataset for object detection, and the detection accuracy and inference speed of CXR-RefineDet have reached 0.1686 mAP and 6.8 fps, respectively. The experimental results show that both the backbone RRNet and the structure Information Reuse can effectively improve the detection accuracy of the network. Through comparison experiments with mainstream object detection algorithms, it is found that the detection accuracy and detection speed of CXR-RefineDet are significantly better than the existing mainstream object detectors under the condition of moderate parameters. In addition, CXR-RefineDet has a good performance between accuracy and speed, which can not only effectively alleviate the problem of high computational resource consumption caused by the use of large models and large resolution in the current lung lesion detection but also provide objective conditions for the actual implementation of the computer-aided diagnosis system.

## Figures and Tables

**Figure 1:** Comparison of the proposed CXR-RefineDet and other mainstream object detectors. CXR-RefineDet at 512 resolution reaches 0.1686 mAP, surpassing all mainstream detectors, and its single image inference speed is nearly 2 times that of other detectors.

**Figure 2:** Architecture structure of CXR-RefineDet.

**Figure 3:** The architecture of different blocks: (a) RepVGG block and (b) Resblock.

**Figure 4:** Comparison of VGG-16, ResNet-34, and the backbone RRNet we designed. (a) VGG-16. (b) RRNet. (c) ResNet-34.

**Figure 5:** The connection method of the original RefineDet network output layer and the improved Information Reuse.

**Figure 6:** Distribution of various lesion categories in VinDr-CXR dataset.

**Figure 7:** The chest X-ray test results, where (1) is the true label of the VinDr-CXR dataset, (2) and (3) are the comparison images of the test results of RefineDet and CXR-RefineDet on the VinDr-CXR test set, respectively, and the target boxes of the same color represent the same lesion category.

**Table 1:** Performance comparison of different backbone networks.

Backbone	mAP	Params (*M*)

All-Resblock	0.1521	49.98
All-RepVGG block	0.1513	35.15
ResNet-18	0.1409	30.16
ResNet-34	0.1525	40.26
REVGG-A0	0.1374	**23.52**
REVGG-A1	0.1409	29.77
REVGG-B0	0.1434	30.23
REVGG-B1	0.1488	72.05
RRNet (ours)	**0.1572**	49.76

**Table 2:** Effectiveness of various designs.

Component	Chest-X_ray RefineDet					

VGG Pretraining model				√		
Batch normalization	√	√	√			
Information Reuse	√	√				
RRNet	√					
mAP	**0.1686**	0.1587	0.1515	0.1514		0.1173

**Table 3:** Detection results of different methods on VinDr-CXR test set.

Method	Backbone	Input size	mAP	Inference speed (fps) w/o reparam	Params (*M*)

RetinaNet	ResNet-50	512 × 512	0.1269	3.7	36.37
	ResNet-101		0.1494	3.5	55.37

Faster RCNN	ResNet-50	512 × 512	0.1597	3.7	41.19
	ResNet-101		0.1569	3.5	60.18

GA-Faster RCNN	ResNet-50	512 × 512	0.1464	3.3	41.78

Cascade RCNN	ResNet-50	512 × 512	0.1512	3.3	68.97
	ResNet-50-DCN		0.1613	3.2	69.55
	ResNet-101		0.1631	3.1	87.96
	ResNet-101-DCN		0.1560	3.0	89.24

VFNet	ResNet-50	512 × 512	0.1413	3.6	32.51
	ResNet-101		0.1505	3.4	51.51

ATSS	ResNet-50	512 × 512	0.1478	3.7	31.92
	ResNet-101		0.1538	3.5	50.91

RefineDet	VGG-16	320 × 320	0.1149	10.8	—
RefineDet	VGG-16	512 × 512	0.1173	9.9	33.51
CXR-RefineDet (ours)	RRNet	320 × 320	0.1392	9.6	—
CXR-RefineDet (ours)	RRNet	512 × 512	0.1618	6.8	49.76

## Data Availability

The datasets used and analyzed during the current study are available from the corresponding author upon reasonable request.

## References

[1] Zhang Y., Wang S., Zhao H., Guo Z., Sun D. (2021). CT image classification based on convolutional neural network. *Neural Computing and Applications*.

[2] Matsumoto T., Doi K., Kano A., Nakamura H., Nakanishi T. (1993). Evaluation of the potential benefit of computer-aided diagnosis (CAD) for lung cancer screenings using photofluorography: analysis of an observer study. *Nippon Igaku Hoshasen Gakkai Zasshi*.

[3] Wang H., Li X., Jhaveri R. H. (2021). Sparse Bayesian learning based channel estimation in FBMC/OQAM industrial IoT networks. *Computer Communications*.

[4] Wang Z., Jiang X., Liu J., Cheng K.-T., Yang X. (2020). Multi-task siamese network for retinal artery/vein separation via deep convolution along vessel. *IEEE Transactions on Medical Imaging*.

[5] Tariq J. A., Ben I. A., Abdel K. S. (2021). Tumor edge detection in mammography images using quantum and machine learning approaches. *Neural Computing and Applications*.

[6] Girshick R., Donahue J., Darrell T., Malik J. Rich feature hierarchies for accurate object detection and semantic segmentation.

[7] Zhao M., Wang H., Han Y. (2020). SEENS: nuclei segmentation in Pap smear images with selective edge enhancement. *Future Generation Computer Systems*.

[8] Setio A. A. A., Ciompi F., Litjens G. (2016). Pulmonary nodule detection in ct images: false positive reduction using multi-view convolutional networks. *IEEE Transactions on Medical Imaging*.

[9] Ronneberger O., Fischer P., Brox T. U-net: convolutional networks for biomedical image segmentation.

[10] Rocha J., Cunha A., Mendonça A. M. (2020). Conventional filtering versus U-Net based models for pulmonary nodule segmentation in CT images. *Journal of Medical Systems*.

[11] Zhao Z. Q., Zheng P., Xu S. T., Wu X. (2018). Object detection with deep learning: a review. *IEEE Transactions on Neural Networks and Learning Systems*.

[12] Kim E., Kim S., Seo M., Yoon S. XProtoNet: diagnosis in chest radiography with global and local explanations.

[13] Girshick R. Fast R-CNN.

[14] Li X., Shen L., Xie X. (2019). Multi-resolution convolutional networks for chest X-Ray radiograph based lung nodule detection. *Artificial Intelligence in Medicine*.

[15] He K., Gkioxari G., Dollar P., Girshick R. Mask R-CNN.

[16] Yan K., Peng Y., Sandfort V., Bagheri M., Lu Z. RM summers holistic and comprehensive annotation of clinically significant findings on diverse CT images: learning from radiology reports and label ontology.

[17] Liang J., Ye G., Guo J., Huang Q., Zhang S. (2021). Reducing false-positives in lung nodules detection using balanced datasets. *Frontiers in Public Health*.

[18] Xiao Y., Wang X., Li Q. (2021). A cascade and heterogeneous neural network for CT pulmonary nodule detection and its evaluation on both phantom and patient data. *Computerized Medical Imaging and Graphics*.

[19] Lin T. Y., Dollar P., Girshick R. Feature pyramid networks for object detection.

[20] Lin T. Y., Goyal P., Girshick R., He K. M., Dollar P. (2017). Focal loss for dense object detection. *IEEE Transactions on Pattern Analysis and Machine Intelligence*.

[21] He K., Zhang X., Ren S., Sun J. Deep residual learning for image recognition.

[22] Jie H., Li S., Gang S., Albanie S. Squeeze-and-excitation networks.

[23] Nguyen H., Lam K., Le L. T. (2012). VinDr-CXR: an open dataset of chest X-rays with radiologist’s annotations. https://arxiv.org/abs/2012.15029.

[24] Zhang S., Wen L., Bian X., Lei Z., Li S. Z. Single-shot refinement neural network for object detection.

[25] Simonyan K., Zisserman A. (2014). Very deep convolutional networks for large-scale image recognition. https://arxiv.org/abs/1409.1556.

[26] Huang G., Liu Z., Der Maaten L., Weinberger K. Q. Densely connected convolutional networks.

[27] Xie S., Girshick R., Dollár P., Tu Z., He K. Aggregated residual transformations for deep neural networks.

[28] Zhang H., Wu C., Zhang Z. (2020). Resnest: splitattention networks. https://arxiv.org/abs/2004.08955.

[29] Li X., Wang W., Hu X., Yang J. Selective kernel networks.

[30] Ding X., Zhang X., Ma N., Han J., Ding G., Sun J. RepVGG: making VGG-style ConvNets great again.

[31] Deng J., Dong W., Socher R., Li L., Li K., Li F. Imagenet: a large--scale hierarchical image database.

[32] Zhu R., Zhang F., Wang X., Wen L., Mei T. ScratchDet: training single-shot object detectors from scratch.

[33] Chen Q., Huang M., Wang H., Xu G. (2021). A feature discretization method based on fuzzy rough sets for high-resolution remote sensing big data under linear spectral model. *IEEE Transactions on Fuzzy Systems*.

[34] Everingham M., Eslami S. M. A., Van Gool L., Williams C. K. I., Winn J., Zisserman A. (2015). The pascal visual object classes challenge: a retrospective. *International Journal of Computer Vision*.

[35] Zhang H., Wang Y., Dayoub F., Sünderhauf N. (2020). VarifocalNet: an IoU-aware dense object detector. https://arxiv.org/abs/2004.08955.

[36] Zhang S., Chi C., Yao Y., Lei Z., Li S. Z. Bridging the gap between anchor-based and anchor-free detection via adaptive training sample selection.

